# Inhibition of Lipopolysaccharide-Induced Proinflammatory Responses by *Buddleja officinalis* Extract in BV-2 Microglial Cells via Negative Regulation of NF-κB and ERK1/2 Signaling

**DOI:** 10.3390/molecules18089195

**Published:** 2013-07-31

**Authors:** Won-Jun Oh, Uhee Jung, Hyun-Soo Eom, Hee-June Shin, Hae-Ran Park

**Affiliations:** Radiation Biotechnology Research Division, Advanced Radiation Technology Institute, Korea Atomic Energy Research Institute (KAERI), 1266 Sinjeong-dong Jeongeup-si, Jeonbuk 580-185, Korea; E-Mails: owjmgm@kaeri.re.kr (W.-J.O.); ehsoo@kaeri.re.kr (H.-S.E.); hj-shin@kaeri.re.kr (H.-J.S.); hrpark@kaeri.re.kr (H.-R.P.)

**Keywords:** *Buddleja officinalis*, neuroinflammation, microglia, NF-κB, ERK1/2

## Abstract

*Buddleja officinalis* has been traditionally used in the supportive treatment of inflammatory and neuronal diseases in Korea and China. Although several reports have shown the anti-inflammatory effects of *Buddleja officinalis*, the anti-neuroinflammatory effect has remained unclear. In this study, we aimed to investigate the inhibitory effects of flower buds of *B. officinalis* Maximowicz water extract (BOWE) on LPS-induced inflammatory processes in BV-2 microglial cells. BOWE dose-dependently inhibited the production of nitric oxide as well as iNOS mRNA expression. Moreover, BOWE prevented IL-1β and IL-6 mRNA expression. However, BOWE had no effect on LPS-induced COX-2 or TNF-α mRNA expression. The extract also had no effect on LPS-stimulated p38 MAPK, JNK, and c-Jun phosphorylation, whereas ERK1/2 phosphorylation was strongly inhibited by BOWE. BOWE also inhibited the LPS-induced degradation of IκB-α, and LPS-induced phosphorylation of p65 NF-κB protein. These data indicate that BOWE inhibited the nitric oxide production and pro-inflammatory gene expression in BV-2 microglial cells, possibly through a negative regulation of the NF-κB and ERK1/2 pathways. Further identification of the direct target molecule(s) of BOWE is required to support its use as an anti-neuroinflammatory agent against the neurodegenerative disorders.

## 1. Introduction

Inflammation plays a major role in the pathology of neurodegenerative diseases [1,2]. In the central nervous system (CNS), inflammation is dependent on the secretion of various inflammatory substances by resident macrophages such as microglia [1,2,3,4]. The activation of microglia is one of the hallmarks and driving forces of brain inflammation, which is believed to cause inflammation-induced neuronal cell death in a number of neurodegenerative diseases, including Parkinson’s disease [4], Alzheimer’s disease [5,6], prion diseases [6], and multiple sclerosis [7]. Although microglia have been reported to promote neuronal cell viability and survival in several studies, much evidence indicates that activated microglia exert a negative effect on brain neurogenesis through excessive synthesis and the secretion of various inflammatory mediators such as nitric oxide (NO), interleukin-6 (IL-6), tumor necrosis factor-α (TNF-α), and IL-1β [2,4].

The activation of microglia is mediated by various transcription factors and protein kinases. In microglia stimulated by lipopolysaccharide (LPS), toll-like receptors are activated and give rise to the nuclear factor-κB (NF-κB) and activating protein 1 (AP-1) signaling and the releases of pro-inflammatory molecules such as NO, cytokines, and chemokines [8,9,10]. The mitogen-activated protein kinase (MAPK) pathway is related to AP-1 signaling, which mediates pro-inflammatory gene expression during LPS-induced microglial activation. The phosphorylation and activation of p38 MAPK, extracellular signal-regulated kinase (ERK), and c-Jun NH_2_-terminal kinase (JNK) has been demonstrated in immune cells by various inflammatory stimuli [10,11]. NF-κB is also a transcription factor involved in the inflammatory process, which is activated by phosphorylation of IκB subunit and its dissociation from the inactive cytoplasmic complex, followed by the translocation of active dimer of p50 and p65 to the nucleus [12]. The regulation of these microglial activation and CNS inflammatory responses may be one of the promising therapeutic strategies for various neurodegenerative diseases.

*Buddleja officinalis* Maximowich (Loganiaceae) has been used to treat strokes, headaches, vascular diseases, diabetes, and neurological disorders in traditional Korean medicine [13]. *B. officinalis* contains terpenoids, flavonoids, phenylethanoids, and saponins such as methylcatalpol, betulalbusides, apigenin, isorhoifolin, linarin, salidroside, acteoside, echinacoside, and buddlejasaponin [14]. Various reports have shown that the components like apigenin and linarin have a protective effect against oxidative stress, inflammation and neuronal disorder [15,16,17]. However, the pharmacological studies on *B. officinalis* are limited, and the detailed mechanism of its anti-inflammatory activity is largely unknown [18]. Therefore, in order to study the neuroprotective mechanism of *B. officinalis*, we examined its inhibitory effects on pro-inflammatory mediators and cytokine mRNA expression profiles as well as the underlying signaling pathways in BV-2 murine microglia cells, which are frequently used in microglial function studies. We demonstrated in this study that *B. officinalis* water extract (BOWE) inhibited LPS-induced NO release, and iNOS, IL-1β, and IL-6 expression, but showed no effects on LPS-induced COX-2 and TNF-α expression in BV-2 cells, and that the anti-inflammatory effects of BOWE were exerted by the regulation of ERK 1/2 and NF-κB signaling pathways.

## 2. Results and Discussion

### 2.1. BOWE Attenuates LPS-Induced NO Production

We first examined the suppressive effect of *B. officinalis* water extract (BOWE) on LPS-induced NO production in BV-2 microglia cells. LPS stimulation strongly increased the NO production in BV-2 microglial cells (Figure 1A). However, pretreatment of BV-2 cells with BOWE at 50–200 µg/mL significantly inhibited the LPS-induced NO production in a dose-dependent manner (Figure 1A). These effects of BOWE were not due to cytotoxicity since BOWE at these concentrations did not show any significant reduction in cell viability (Figure 1B).

**Figure 1:** Effect of BOWE on LPS-induced NO (**A**) and cell viability assay (**B**): BV-2 cells were pretreated with or without the indicated doses of BOWE for 4 h and then stimulated with LPS (0.1 μg/mL) for 18 h. The culture supernatants were subsequently collected and analyzed for nitrite levels. The cell viability was determined by CCK assay. Data are presentedas the means ± SEM of triplicates from separate experiments. * *p* < 0.05 and ** *p* < 0.01 denote significant differences compared to the group treated with LPS only.

### 2.2. BOWE Inhibits LPS-Induced iNOS Expression, but not COX-2 Expression

Next, we determined the iNOS and COX-2 mRNA expressions using RT-PCR to understand the anti-inflammatory mechanism of BOWE. LPS-stimulated BV-2 cells showed elevated levels of iNOS or COX-2 mRNA when compared with non-stimulated cells (Figure 2). BOWE treatment (50, 100, and 200 µg/mL) attenuated the iNOS mRNA expression level in LPS-stimulated BV-2 cells in a dose-dependent manner (Figure 2A). However, BOWE did not affect LPS-induced COX-2 expression (Figure 2B). These results show that BOWE inhibited NO release by suppressing iNOS mRNA expression, but did not affect COX-2 mRNA expression in LPS-stimulated microglial cells.

NO is generated in different cell types by three isoforms of NOS and is carefully regulated to maintain homeostasis [19,20,21]. iNOS, one of the NOS isoforms, is a key enzyme in inflammatory processes [21]. High levels of NO produced by iNOS under pathological conditions, such as inflammatory diseases, are associated with atherosclerosis, cancer, and neurodegenerative diseases [19,20,21]. Thus, it might be beneficial in therapy for CNS inflammatory and neurodegenerative diseases to down-regulate iNOS expression and/or to reduce the level of NO generated in response to inflammatory stimuli in microglia. Our findings indicate that BOWE inhibited iNOS mRNA expression and subsequent NO release, suggesting its possible protective effects against neuroinflammation in BV-2 microglia cells. However, BOWE inhibited LPS-induced iNOS activity without any effect on COX-2 expression (Figure 2). Accordingly, these data suggest that BOWE exerts selective anti-inflammatory effects by down-regulating iNOS expression but not COX-2 expression.

**Figure 2:** Effect of BOWE on LPS-induced mRNA expression levels of iNOS and COX-2 in BV-2 cells: For mRNA expression, BV-2 cells were pretreated with BOWE for 4 h and then stimulated with LPS (0.1 μg/mL) for 18 h. Total RNA was isolated, and mRNA levels of iNOS (A) and COX-2 (B) were then measured by RT-PCR. β actin expression was used as an internal control. The quantification of relative band intensities from three independent experiments were analyzed by densitometry and expressed as means ± SEM. * *p* < 0.01 denotes a significant difference compared to the group treated with LPS only.

### 2.3. BOWE Inhibits LPS-Induced IL-1β and IL-6, but not TNF-α

Excessive pro-inflammatory cytokines, such as TNF-α, IL-1β, and IL-6, are produced by microglia in the brain, which are suspected to be associated with brain inflammation, neurodegeneration, and many neurological disorders [1,2,4,5,6,7]. There are many evidences that activated microglia suppress neurogenesis by affecting the neural stem or progenitor cells via pro-inflammatory cytokine production [1]. Therefore, we next examined whether BOWE can inhibit the production of LPS-induced pro-inflammatory cytokines including IL-1β, IL-6, and TNF-α.

LPS-stimulated BV-2 cells showed significant increases in IL-1β, IL-6, and TNF-α mRNA levels. As shown in Figure 3A,B, BOWE had inhibitory effects on IL-1β and IL-6 mRNA expression in a dose-dependent manner. However, treatment with BOWE did not attenuate TNF-α mRNA expression in LPS-activated BV-2 cells (Figure 3C). Also when the secreted protein levels were examined, IL-6 secretion was inhibited by the pretreatment with BOWE in a dose-dependent manner, but TNF-α secretion was not affected by BOWE (Figure 4A,B). Our findings that BOWE suppressed IL-1β and IL-6 but did not affect TNF-α (Figure 3C, Figure 4A) and COX-2 (Figure 2B) suggested that BOWE can suppress the NF-κB pathway but not the AP-1 pathway since it has been previously reported that IL-6 production is mediated by NF-κB activation [22] but COX-2 and TNF-α production is closely related with activation of AP-1 signaling [23,24,25].

**Figure 3:** Effect of BOWE on the mRNA expressions of IL-1β (**A**), IL-6 (**B**), and TNF-α (**C**): BV-2 cells were pretreated with or without the indicated concentrations of BOWE for 4 h and then stimulated with LPS (0.1 μg/mL) for 18 h. Total RNA was isolated and mRNA expressions of the aforementioned cytokines were measured by RT-PCR. β actin was used as a housekeeping gene. The quantification of relative band intensities from three independentexperiments were analyzed by densitometry and expressed as means ± SEM. * *p* < 0.01denotes a significant difference compared to the group treated with LPS only.

**Figure 4:** Effect of BOWE on LPS-induced TNF-α (**A**) and IL-6 (**B**) release: BV-2 cells were pretreated with or without the indicated concentrations of BOWE for 4 h and then stimulated with LPS (0.1 μg/mL) for 18 h. The culture supernatants were subsequently harvested and analyzed for TNF-α and IL-6 levels by ELISA. Data are presented as the means ± SEM in each group (n = 3). * *p* < 0.05 and ** *p* < 0.01 denote significant differences compared to the group treated with LPS only.

### 2.4. BOWE Inhibits LPS-Induced NF-κB Signaling

Next, we investigated the repressive effect of BOWE on NF-κB activation in BV-2 cells. LPS markedly decreased the IκB-α level and increased the phosphorylation of IκB-α and NF-κB p65 subunit compared with those in non-stimulated BV-2 cells suggesting the activation of NF-κB (Figure 5). However, the pretreatment with BOWE effectively blocked the IκB-α degradation and the phosphorylation of IκB-α and p65. These results indicate that BOWE inhibited the NF-κB activation in LPS-stimulated BV-2 cells.

Several studies have demonstrated that IKK/NF-κB and c-Jun/AP-1 are the two major cellular pathways involved in LPS-induced microglial activation processes, which modulate iNOS expression and orchestrate inflammation-associated gene expression [3,23]. Activation of NF-κB is typically involved in IκB phosphorylation by the IκB kinase complex, which results in IκB degradation and the translocation of p50/p65 NF-κB to the nucleus [12]. In the present study, BOWE inhibited LPS-induced IκB-α phosphorylation and reversed LPS-mediated IκB-α degradation (Figure 5). Furthermore, BOWE also suppressed LPS-stimulated p65 NF-κB phosphorylation in BV-2 cells (Figure 5). These findings suggest that the transcriptional down-regulation of the expression of iNOS and several inflammatory mediators such as IL-1β and IL-6 by BOWE results from an inhibition of the NF-κB signaling pathway.

**Figure 5:** Effect of BOWE on IκB-α and NF-κB p65 phosphorylation in LPS-stimulated BV-2 cells: BV-2 cells were pretreated with or without the indicated concentrations of BOWE for 4 h and then stimulated with LPS (0.1 μg/mL) for 18 h. The cellular proteins from the cells were used for the detection of phosphorylated forms of IκB-α and NF-κB p65 by western blotting. β-actin was used as a loading control.

### 2.5. BOWE Inhibits LPS-Induced ERK1/2 Phosphorylation, but not p38 and JNK Phosphorylation

The variety of stimuli activating NF-κB also activate MAPKs, which in turn activate other transcription factors such as AP-1 on glial cells [9,23]. Three major subfamilies of MAPK cascades, *i.e.*, ERK1/2, JNK1/2, and p38 MAPK, have been defined [10,11]. Therefore, to assess whether the MAPK pathways are involved in the repressive effect of BOWE on the release of pro-inflammatory mediators, we examined the phosphorylation of ERK1/2, p38 MAPK, and JNK in LPS-stimulated BV-2 cells. We also investigated whether BOWE can inhibit c-Jun phosphorylation to demonstrate a connection with AP-1 signaling. As expected, LPS treatment remarkably elevated the phosphorylation of ERK1/2, p38, JNK, and c-Jun. However, BOWE treatment showed the differential effects on LPS-induced phosphorylation of these proteins. The phosphorylation of ERK1/2 was remarkably attenuated by BOWE, but the phosphorylation of p38 MAPK, JNK, or c-Jun was not affected by BOWE (Figure 6). These results indicate that BOWE strongly blocked the ERK1/2 pathway but not p38 and JNK pathways in LPS-stimulated BV-2 cells.

**Figure 6:** Effect of BOWE on MAPK phosphorylation in LPS-stimulated BV-2 cells: BV-2 cells were pretreated with or without the indicated concentrations of BOWE for 4 h and then stimulated with LPS (0.1 μg/mL) for 18 h. The cellular proteins from the cells were used for the detection of phosphorylated or total forms of ERK1/2, p38 MAPK, JNK1/2, and c-Jun by western blotting.

Several studies have shown that the ERK1/2 pathway is different from other MAPK pathways such as JNK and p38 MAPK in various inflammatory reactions [22,23,26,27,28]. For example, one report showed that *Streptococcus mutans*-induced TNF-α expression is inhibited by treatment with SB203580, a p38 MAPK inhibitor, or SP600125, a JNK inhibitor, whereas IL-1β expression is restrained by pretreatment with a ERK/p38/JNK inhibitor [26]. Another report showed a similar result that leptin enhances LPS-induced TNF-α production in Kupffer cells through the JNK and p38 MAPK pathways, but not ERK [27]. These reports indicate that JNK and p38 MAPK, but not ERK, are involved in the TNF-α and COX-2 expression. However, ERK1/2 is suggested to be an upstream signal of NF-κB, which regulates IL-6 production in activated microglia [22]. The inflammatory signaling pathways based on these reports are illustrated in Figure 7. Our results clearly demonstrated that BOWE down-regulated NF-κB activation and ERK1/2 phosphorylation with subsequent suppression of NO, iNOS, IL-1β, and IL-6. But BOWE did not affect JNK, p38 MAPK, and AP-1 activation. These results suggest that BOWE inhibited LPS-induced inflammatory responses in BV-2 microglia cells by selectively targeting ERK1/2 and NF-κB signal pathways (Figure 7). Further identification of the direct target molecule(s) of BOWE is required to support its use as an anti-neuroinflammatory agent against the neurodegenerative disorders.

**Figure 7:** Suggested anti-inflammation mechanism of BOWE in LPS-treated BV-2 cells: In BV-2 cells treated with LPS, BOWE prevented the activation of ERK1/2 and NF-κB, and subsequently attenuated the production of IL-6, IL-1β, iNOS, and nitric oxide. BOWE did not have any effect on the activation of JNK, p38, and c-Jun and the production of TNF-α and COX-2. The negative regulation of ERK1/2 and NF-κB activation is supposed to be the main mechanism of anti-inflammatory action of BOWE in BV-2 cells.

## 3. Experimental

### 3.1. Preparation of B. officinalis Water Extract

The flower buds of *B. officinalis* Maximowicz which were collected from Sichuan in China were purchased from the Medical Material Company (Dukhyundang, Seoul, Korea). Dried *B. officinalis* (100 g) was boiled in 1.5 liters of purified water for 150 min at 100°C, filtered through Whatman No. 2 paper, and then concentrated in a rotary vacuum evaporator (Eyela, Model N-11, Tokyo, Japan). The concentrated extract was lyophilized (Ilshin, model FD5505, Seoul, Korea) to produce a powder and then stored at −20 °C until use. The 6.92 g of lyophilized powder was obtained from 100 g of dried *B. offininalis*.

### 3.2. Cell Culture

BV-2 cells were kindly provided by Prof. S.H. Han at the School of Dentistry, Seoul National University. BV-2 cells were cultured in Dulbecco’s modified Eagle medium (DMEM) (Hyclone Co., Logan, UT, USA) supplemented with 5% heat-inactivated fetal bovine serum (Hyclone), 100 µg/mL streptomycin, and 100 U/mL penicillin (Sigma-Aldrich, St. Louis, MO, USA) in a humidified atmosphere of 5% CO_2_ at 37 °C.

### 3.3. Cell Viability and NO Assay

A cell viability assay was performed using an EZ-Cytox Cell Viability Assay kit (Daeillab Service Co., Seoul, Korea) to check the cytotoxic effect of BOWE. BV-2 cells were plated in 96-well plates at 3 × 10^3^ cells/well and pretreated with or without BOWE (50, 100, and 200 µg/mL) for 4 h. After an 18 h LPS (0.1 µg/mL) stimulation, EZ-Cytox was added to the cells for 1 h in a humidified atmosphere of 5% CO_2_ at 37 °C, and the absorbance was measured at 450 nm using a microplate reader (Molecular Devices, Sunnyvale, CA, USA). To determine the NO production, BV-2 cells (2 × 10^5^ cells/mL) were plated on a 100 mm plate and pretreated with or without BOWE (50, 100, and 200 µg/mL) for 4 h. After LPS (0.1 µg/mL) stimulation for 18 h, the nitrite levels were measured in cell culture supernatants based on the Griess reaction (Sigma-Aldrich) and compared with a nitrite standard curve. The absorbance was measured at 540 nm.

### 3.4. Enzyme-Linked Immunosorbent Assay (ELISA)

BV-2 cells (2 × 10^5^ cells/mL) were treated with different BOWE concentrations. The BV-2 cell supernatant was collected at 18 h after LPS stimulation, and the levels of cytokines including TNF-α and IL-6 were measured in a cultured medium using commercially available OptEIA kits (BD Biosciences, San Diego, CA, USA) according to the manufacturer’s instructions. Briefly, the serial dilutions of the protein standards and samples were added to 96-well ELISA plates, followed by biotinylated anti-TNF-α or IL-6 detection antibodies. After washing with 0.05% PBST, a SAv-HRP solution was added followed by a TMB substrate solution. The reaction was stopped using a stop solution. The optical density was detected at ref 450–570 nm using a microplate reader (Molecular Devices). The concentration of each sample was calculated from a linear equation derived from the standard curve of known cytokine concentrations.

### 3.5. RNA Isolation and Reverse Transcription-Polymerase Chain Reaction (RT-PCR)

Cultured BV-2 murine microglia (2 × 10^5^ cells/mL) were pre-incubated alone or with BOWE for 4 h and then stimulated with LPS for 18 h. The total RNA was isolated using Easy-BLUE kits (iNTRON Biotechnology, Seoul, Korea) according to the manufacturer’s instructions and stored at −70 °C until use. Briefly, 5 µg RNA was annealed with poly(dT) for 5 min at 70 °C and cooled for 5 min on ice, reverse transcribed using an RT mixture (dNTP, 5× RT buffer, RTase) with 10 µL of a reaction mixture, and run for 60 min at 42°C in a water bath. The reactions were terminated at 95 °C for 5 min to inactivate the reverse transcriptase. RT-PCR was performed using aliquots of cDNA obtained from the RT reaction in a PCR mixture (dNTP, Taq polymerase, Taq buffer). PCR products were electrophoresed in a 1% agarose gel stained with ethidium bromide and visualized using a Digital Gel Image system (EDAS 290; Kodak, Rochester, NY, USA). The band intensities for iNOS, COX-2, TNF-α, IL-1β, and IL-6 mRNA expression levels were normalized to the corresponding β-actin band, which is a housekeeping gene used as an RNA internal standard, and the ratios were compared. The primers used for the RT-PCR are shown in Table 1.

**Table 1:** Primer sequences used for RT-PCR.

iNOS [29]	sense	CCG TCC ACA GTA TGT GAG GA
	anti-sense	GAA CTC CAA GGT GGC AGC A
COX-2 [30]	sense	TGA TGA CTG CCC AAC TCC CAT G
	anti-sense	AAT GTT GAA GGT GTC CGG CAG C
TNF-α [30]	sense	CAG ACC CTC ACA CTC AGA TCA TCT T
	anti-sense	CAG AGC AAT GAC TCC AAA GTA GAC CT
IL-1β [31]	sense	GAG GCT GAC AGA CCC CAA AAG AT
	anti-sense	GCA CGA GGC ATT TTT GTT GTT CA
IL-6 [22]	sense	GGA GCC CAC CAA GAA CGA TAG TCA
	anti-sense	GAA GTA GGG AAG GCC GTG GTT

### 3.6. Western Blot Analysis of c-Jun, MAPKs, and NF-κB Protein Expression

BOWE-treated and untreated BV-2 cells were scraped and washed twice with an ice-cold phosphate-buffered saline. The washed cell pellets were lysed in a PRO-PREP Protein Extraction Solution (iNtRON Biotechnology). The protein was then measured using a BCA Protein Assay kit (Pierce Biotechnology, Rockford, IL, USA). Equal amounts of protein (20 µg) were boiled with 1% sodium dodecyl sulfate (SDS) and 1% β-mercaptoethanol for 5 min, separated in a 10% SDS-polyacrylamide gel, and then transferred onto polyvinylidine fluoride membranes. The membranes were incubated with a blocking buffer (5% skim milk in 1× TBST) for 4 h at room temperature and then overnight at 4 °C with primary antibodies. The primary antibodies used were as follows: the phosphor- or total forms of ERK1/2, p38 MAPK, JNK, c-Jun (rabbit polyclonal antibodies, 1:1000, Cell Signaling Technology, Danvers, MA, USA), phosphor-NF-κB (p65) (rabbit polyclonal antibody, 1:1000, Cell Signaling Technology), phosphor IκB-α (rabbit monoclonal antibody, 1:1000, Cell Signaling Technology), total IκB-α (rabbit polyclonal antibody, 1:1000, Cell Signaling Technology), and β-actin (mouse monoclonal antibody, 1:10000, Santa Cruz Biotechnology, Santa Cruz, CA, USA).

### 3.7. Statistical Analysis

The data were analyzed using a one-way analysis of variance, followed by a Dunnett’s test using Statistical Analysis Software, version 9.1 (SAS Institute, Cary, NC, USA). All values are presented as mean ± standard error. *p* < 0.05 was considered significant.

## 4. Conclusions

In summary, our study demonstrated that BOWE influenced the synthesis and release of NO, iNOS, and pro-inflammatory factors including IL-1β and IL-6 by affecting intracellular signal transduction pathways such as ERK 1/2 and the transcription factor NF-κB in BV-2 microglial cells. These findings suggest that further studies on BOWE will lead to a potential therapeutic strategy for treating neurological diseases in which inflammation-stimulated microglia contribute to neurodegeneration.

## References

[1] Whitney N.P., Eidem T.M., Peng H., Huang Y., Zheng J.C. (2009). Inflammation mediates varying effects in neurogenesis: relevance to the pathogenesis of brain injury and neurodegenerative disorders. J. Neurochem..

[2] Liu B. (2003). Role of Microglia in Inflammation-Mediated Neurodegenerative Diseases: Mechanisms and Strategies for Therapeutic Intervention. J. Pharm. Exp. Ther..

[3] Saha R.N., Pahan K. (2006). Regulation of Inducible Nitric Oxide Synthase Gene in Glial Cells. Antioxid. Redox Signal..

[4] Kim Y.S., Joh T.H. (2006). Microglia, major player in the brain inflammation: Their roles in the pathogenesis of Parkinson’s disease. Exp. Mol. Med..

[5] McGeer E.G., McGeer P.L. (2003). Inflammatory processes in Alzheimer’s disease. Prog. Neuro Psychoph..

[6] Eikelenboom P., Bate C., van Gool W.A., Hoozemans J.J.M., Rozemuller J.M., Veerhuis R., Williams A. (2002). Neuroinflammation in Alzheimer’s disease and prion disease. Glia.

[7] Sanders P., de Keyser J. (2007). Janus faces of microglia in multiple sclerosis. Brain Res..

[8] Sabroe I., Dower S.K., Whyte M.K.B. (2005). The Role of Toll-Like Receptors in the Regulation of Neutrophil Migration, Activation, and Apoptosis. Clin. Infect. Dis..

[9] Necela B.M., Su W., Thompson E.A. (2008). Toll-like receptor 4 mediates cross-talk between peroxisome proliferator-activated receptor γ and nuclear factor-κB in macrophages. Immunology.

[10] Kaminska B. (2005). MAPK signalling pathways as molecular targets for anti-inflammatory therapy—From molecular mechanisms to therapeutic benefits. Biochim. Biophys. Acta.

[11] Krens S.F.G., Spaink H.P., Snaar-Jagalska B.E. (2006). Functions of the MAPK family in vertebrate-development. FEBS Lett..

[12] Hayden M.S., Ghosh S. (2008). Shared Principles in NF-κB Signaling. Cell.

[13] Hur J. (1983). Tongeuibokam.

[14] Tai B.H., Nhiem N.X., Quang T.H., Ngan N.T.T., Tung N.H., Kim Y., Lee J.-J., Myung C.-S., Cuong N.M., Kim Y.H. (2011). A new iridoid and effect on the rat aortic vascular smooth muscle cell proliferation of isolated compounds from Buddleja officinalis. Bioorgan. Med. Chem. Lett..

[15] Kim Y.H., Lee Y.S., Choi E.M. (2011). Linarin isolated from Buddleja officinalis prevents hydrogen peroxide-induced dysfunction in osteoblastic MC3T3-E1 cells. Cell. Immunol..

[16] Lou H., Fan P., Perez R.G., Lou H. (2011). Neuroprotective effects of linarin through activation of the PI3K/Akt pathway in amyloid-β-induced neuronal cell death. Bioorgan. Med. Chem..

[17] Wang Y.-C., Huang K.-M. (2013). *In vitro* anti-inflammatory effect of apigenin in the Helicobacter pylori-infected gastric adenocarcinoma cells. Food Chem. Toxicol..

[18] Lee D.H., Ha N., Bu Y.M., Choi H.I., Park Y.G., Kim Y.B., Kim M.Y., Kim H. (2006). Neuroprotective effect of Buddleja officinalis extract on transient middle cerebral artery occlusion in rats. Biol. Pharm. Bull..

[19] Lala P.K., Chakraborty C. (2001). Role of nitric oxide in carcinogenesis and tumour progression. Lancet Oncol..

[20] Naseem K. (2005). The role of nitric oxide in cardiovascular diseases. JMAM.

[21] Pannu R., Singh I. (2006). Pharmacological strategies for the regulation of inducible nitric oxide synthase: Neurodegenerative versus neuroprotective mechanisms. Neurochem. Int..

[22] Kim Y.H., Koh H.K., Kim D.S. (2010). Down-regulation of IL-6 production by astaxanthin via ERK-, MSK-, and NF-kappaB-mediated signals in activated microglia. Int. Immunopharmacol..

[23] Song L., Li J., Hu M., Huang C. (2008). Both IKKα and IKKβ are implicated in the arsenite-induced AP-1 transactivation correlating with cell apoptosis through NF-κB activity-independent manner. Exp. Cell Res..

[24] Medeiros R., Figueiredo C.P., Pandolfo P., Duarte F.S., Prediger R.D.S., Passos G.F., Calixto J.B. (2010). The role of TNF-α signaling pathway on COX-2 upregulation and cognitive decline induced by β-amyloid peptide. Behav. Brain Res..

[25] Ramanan S., Kooshki M., Zhao W., Hsu F.-C., Robbins M.E. (2008). PPARα ligands inhibit radiation-induced microglial inflammatory responses by negatively regulating NF-κB and AP-1 pathways. Free Radic. Bio. Med..

[26] Kim J.S., Kim K.D., Na H.S., Jeong S.Y., Park H.R., Kim S., Chung J. (2012). Tumor necrosis factor-alpha and interleukin-1beta expression pathway induced by Streptococcus mutans in macrophage cell line RAW 264.7. Mol. Oral Microbiol..

[27] Shen J., Sakaida I., Uchida K., Terai S., Okita K. (2005). Leptin enhances TNF-alpha production via p38 and JNK MAPK in LPS-stimulated Kupffer cells. Life Sci..

[28] Svensson C., Part K., Kunnis-Beres K., Kaldmae M., Fernaeus S.Z., Land T. (2011). Pro-survival effects of JNK and p38 MAPK pathways in LPS-induced activation of BV-2 cells. Biochem. Biophys. Res. Commun..

[29] Lee P., Hur J., Lee J., Kim J., Jeong J., Kang I., Kim S.Y., Kim H. (2006). 15,16-dihydrotanshinone I suppresses the activation of BV-2 cell, a murine microglia cell line, by lipopolysaccharide. Neurochem. Int..

[30] Zhou F., Wu J.Y., Sun X.L., Yao H.H., Ding J.H., Hu G. (2007). Iptakalim alleviates rotenone-induced degeneration of dopaminergic neurons through inhibiting microglia-mediated neuroinflammation. Neuropsychopharmacology.

[31] Tocharus J., Khonthun C., Chongthammakun S., Govitrapong P. (2010). Melatonin attenuates methamphetamine-induced overexpression of pro-inflammatory cytokines in microglial cell lines. J. Pineal Res..

